The article "Effectiveness of ivermectin-based multidrug therapy in severely hypoxic, ambulatory COVID-19 patients" was retracted in 2025. Reasons: unreliable results or conclusions; concerns about the data; concerns about the results or conclusions.

# Effectiveness of ivermectin-based multidrug therapy in severely hypoxic, ambulatory COVID-19 patients

**DOI:** 10.2217/fmb-2022-0014

**Published:** 2022-02-09

**Authors:** Sabine Hazan, Sonya Dave, Anoja W Gunaratne, Sibasish Dolai, Robert L Clancy, Peter A McCullough, Thomas J Borody

**Affiliations:** ^1^ProgenaBiome, LLC, 1845 Knoll Dr., Ventura, CA 93003, USA; ^2^North End Advisory, 2451 Cumberland Pkwy SE Ste. 3152, Atlanta, GA 30339, USA; ^3^Centre for Digestive Diseases, 229 Great North Road, Five Dock, NSW, 2046, Australia; ^4^Truth for Health Foundation, Tucson, AZ 85728, USA

**Keywords:** coronavirus, COVID, doxycycline, ivermectin, SARS-CoV-2, zinc

## Abstract

**Aims:** Ivermectin is a safe, inexpensive and effective early COVID-19 treatment validated in 20+ random, controlled trials. Having developed combination therapies for *Helicobacter pylori*, the authors present a highly effective COVID-19 therapeutic combination, stemming from clinical observations. **Patients & methods:** In 24 COVID-19 subjects refusing hospitalization with high-risk features, hypoxia and untreated moderate to severe symptoms averaging 9 days, the authors administered this novel combination of ivermectin, doxycycline, zinc and vitamins D and C. **Results & conclusions:** All subjects resolved symptoms (in 11 days on average), and oxygen saturation improved in 24 h (87.4% to 93.1%; p = 0.001). There were no hospitalizations or deaths, less than (p < 0.002 or 0.05, respectively) background-matched CDC database controls. Triple combination therapy is safe and effective even when used in outpatients with moderate to severe symptoms.

**Clinical Trial Registration:** NCT04482686 (ClinicalTrial.gov)

There is currently a lack of effective treatments for early or ambulatory patients with COVID-19. Patients testing positive are sent home to isolate without specific treatment prescribed. However, there is growing evidence that certain repurposed drugs with good safety profiles, taken early, can significantly improve outcomes and even avoid or delay the need for immune-modulators, antiplatelet/antithrombotic therapy and the administration of oxygen [1].

Among the most extensively studied of such COVID-19 therapeutics is ivermectin (IVM), a drug that has been used safely in 3.7 billion doses worldwide since 1987 [2–4]. Recently, Dr Satoshi Omura, the 2015 Nobel Prize co-laureate for the discovery of IVM, and colleagues comprehensively reviewed studies to date on IVM activity against COVID-19, concluding that the evidence demonstrated such efficacy [4]. IVM used alone has been tested in more than 20 randomized, controlled trials (RCTs) for COVID-19 treatment, with statistically highly significant clinical benefits in almost all of these and an average of 62% reduction in risk of death [5]. Five such studies for IVM treatment of COVID-19 recently published in top-tier medical journals have all shown multiple clinical benefits for IVM versus controls, most of these with high statistical significance on the order of p < 0.002 [6–10]. At much greater than the standard single antiparasite dose of 200 μg/kg, IVM is well tolerated [11,12] and has been used in RCTs for COVID-19 treatment at cumulative doses of 1500 μg/kg [13] and 3000 μg/kg [14,15] over 4 or 5 days either without or with mild and transient adverse effects. Not surprisingly, IVM has become extensively used in the prevention and early disease management of COVID-19, particularly in non-Western countries.

Despite this strong evidence of clinical benefit in COVID-19 for IVM therapy, variation in therapeutic regimens, especially with respect to the addition of a broad-spectrum antibiotic and zinc, has led to confusion as to how best to manage acute infections. Indeed, the most impressive of the early ambulatory multidrug therapies, claiming 87% and 75% reductions in hospitalization and deaths, respectively, both with a p-value of 0.001, in 869 high-risk subjects, left optimal management strategy unclear due to a mixed use of IVM and hydroxychloroquine (HCQ) [15]. There is an immediate need for an effective, safe and practically available combination therapy formulation based on the best available data.

At a cellular level, IVM modulates communication between the cytoplasm and nucleus, creating a hostile environment for assemblage of the virus while reducing cytokine-mediated inflammation. In addition, IVM inhibits pathology following infection with the COVID-19 virus, by specifically blocking the binding of the virus ‘spike’ protein to the ACE2 receptor. Finally, IVM has been associated with favorable changes in cellular innate immunity [16].

The authors' group has been systematically developing antiviral drug combinations for COVID-19 and found IVM to be particularly effective as a co-therapy for use early in COVID-19 to shorten the time to symptom resolution and to prevent hospitalization. IVM used alone can at times be only partially effective but not curative [1,6,17]. Thus, the authors chose a combination of safe and widely available medications, approved for other indications and without drug–drug interactions or QT prolongation and one that inhibits intracellular virus replication and possesses some anti-inflammatory properties.

The use of combination therapy for intracellular bacterial infections is not new and has been used successfully to treat tuberculosis, *Helicobacter pylori* (*H. pylori*) infections, leprosy and intracellular viral infections such as hepatitis B and C, in which a single component of the combination therapies is rarely curative. In some viral infections such as HIV, even combined multiple antiviral drugs cannot completely cure but suppress the viral load perpetually [18]. IVM is best known for its broad-spectrum efficacy for parasite infections, its high cure rate and its limited drug resistance when used in combination [19]. Although useful, IVM alone is not the ‘magic bullet’. Combinations can help lower individual doses and reduce side effects. To cover all age group requirements, the authors combined IVM with doxycycline and zinc as active components and with vitamins D and C as replacement ‘excipients’ given to supplement common clinical deficiencies in the aged.

This study reports the use of the above combination therapy in consecutive, ambulatory, complex and at times profoundly hypoxic patients who insisted on avoiding hospitalization and whose oxygen saturation (SpO_2_) was as low as 73%. Participants were treated by an experienced clinical trials team running a trial called Combination Therapy to Treat COVID-19 Infection.

## Methods

### Subjects

Subjects were identified from patients referred by physicians or word-of-mouth in Los Angeles, Ventura County, CA, and other states in the USA. These patients were referred to participate in clinical trials under clinicaltrial.gov ID NCT04482686 (which is a double-blind RCT). However, some did not qualify for this trial, as their SpO_2_ was less than 90%, and were deemed too sick to enter a placebo-controlled trial. All subjects refused hospitalizations for different reasons, including not wanting to die in the hospital. Given subjects were excluded from other studies and refused to go to the hospital, they were treated off-label via telemedicine, during August 2020 and February 2021. Subjects were given the opportunity to participate in this open-label trial with institutional review board (IRB) oversight once the diagnosis was made via swab reverse transcription quantitative real-time PCR (RT-qPCR) testing. Inclusion criteria were as follows: positive PCR for COVID-19, informed consent, age ≥18 years old and agreement to practice two highly effective methods of birth control if of childbearing potential. Exclusion criteria were allergies or drug interactions with the combination therapy components; listed comorbidities, including seizure risk; and pregnancy.

### Treatment

Treatment began as soon as practical, within 72 h of patients presenting to Ventura Clinical Trials. All screened subjects met the inclusion criteria and were enrolled consecutively. Treatment was defined as ‘IVM Combination Therapy’ (ICT) and consisted of 10 days of oral doxycycline (100 mg twice a day), IVM (12 mg on day 1, day 4 and day 8), zinc (25 mg twice a day), vitamin D3 (1500 IU twice a day) and vitamin C (1500 mg twice a day). ICT was given daily for 10 days only.

Two patients (#10 and #23) received an initial treatment on day 1 of 36 mg IVM (rather than 12 mg) due to particularly low SpO_2_ or expected clinical need.

### Monitoring

Subjects self-recorded symptoms in their daily logs (Supplementary Figure 1) for the first 10 days. Electrocardiograms (EKGs), blood pressure, temperature (reported in °F) and SpO_2_ were collected via provided medical equipment at home. On days 1, 5, 10 and 30, SARS-CoV-2 testing swabs were self-collected by subjects and sent to pathology for testing. Pregnancy tests were performed as appropriate.

### End points

End points were time from presentation to negative SARS-CoV-2 PCR, time from presentation to symptom resolution, progression to hospitalization and patient survival.

### Externally controlled trial arm

Given the challenges for COVID-19 of enrolling high-risk, severely hypoxic patients in an open-label trial with an untreated control arm, the treated group arm survival was compared with the control group survival rate in the general population. This externally controlled trial (ECT), also known as a synthetic control arm, was calculated from the public CDC database of COVID-19 subjects [20]. Available information includes age range, presence of any chronic condition (COVID-19 vulnerability or otherwise, conditions not specified), date of infection and whether the COVID-19 diagnosis was laboratory confirmed. The authors used information from all subjects who met the following criteria: age 50+ years old; laboratory-confirmed COVID-19 diagnosis; death/survival, race and sex status available and known; infection prior to March 2021; and any comorbidities. This synthetic control arm data selection was carried out after the authors' data were obtained, to more closely match their subjects, all of whom had some comorbidity and the majority were over 50 years of age. The CDC database was analyzed using CSViewer version 1.3 (EasyMorph, Inc., ON, Canada, http://easymorph.com).

### Covidex calculations & statistics

Covidex and Covidex-F are ambulatory SARS-CoV-2 infection disease severity measures that the authors developed and validated in this study. They are weighted particularly to emphasize SpO_2_, and Covidex-F includes a variable for body temperature.

Covidex score = 1 point (pt) (if history of sleep apnea) + 1 pt (if history of chronic obstructive pulmonary disease [COPD]) + 1 pt (if history of cardiovascular disease) + 1 pt (if history of asthma) + 1 pt (if history of prior clots, ischemia or stroke) + 1 pt (if obese, that is, BMI between ≥30 kg/m^2^ and <40 kg/m^2^) + 2 pts (if severely obese, that is, BMI ≥40) + 1 pt (if age ≥60 years old) + (95-[SpO_2_ as a percentage]) pts. For instance, a hypothetical patient with a history of asthma and morbid obesity with an SpO_2_ prior to treatment of 85% would have a Covidex score of 1 (for asthma) + 2 (for obesity) + 10 (for SpO_2_ of 85%) = 13 pts. Covidex-F score = Covidex score + 1 pt (if temperature on presentation between 99.5°F and 100.4°F) + 2 pts (if temperature on presentation between 100.4°F and 103.5°F) + 3 pts (if temperature on presentation ≥103.5°F).

Best-fit lines were made to assess the correlation between Covidex scores and time from treatment to symptom resolution. Regression was carried out in Prism version 8 (GraphPad Prism software for Windows, CA, USA, www.graphpad.com) using least square regression without weighting or special handling of outliers. All graphs were prepared by and statistical analysis was done using GraphPad Prism version 8, and the error bars are indicative of the standard error of the mean (SEM).

## Results

Table 1 lists all subjects in the study, two of whom did not consent to ICT treatment (subjects #10 and #26, n = 26; n = 24 consenting to treatment), and their associated race, gender, symptoms and fever and other clinical notes. All subjects had COVID-19-related symptoms on presentation, and the symptom range was broad, with several showing shortness of breath (SOB). The vast majority of subjects, 21 of 24 (87.50%), had fever on presentation with a mean temperature for all 24 subjects of 101.2 ± 0.32°F. Specifically, 1/24 (4.17%) had low-grade fever (99.5–100.4°F), 18/24 (75.00%) had medium-grade fever (100.5–103.4°F) and 2/24 (8.33%) had high-grade fever (≥103.4°F).

**Table 1.** Listing of subjects and COVID-associated symptoms on presentation and other characteristics.

ID	Age (years)	Race	Gender	Symptoms	Temp (°F)	O_2_% sat.	O_2_% sat. post 24 h	Rx start date	Symptom resolution date	PCR pos. date	PCR neg. date
1	66	Caucasian	M	Runny nose, sore throat, dizzy, low energy	99.3	90	94	12/14/20	12/21/20	11/6/20	1/17/21
2	62	Caucasian	M	SOB, chest congestion, productive cough, nausea, vomiting	105	77	87	12/8/20	12/18/20	11/30/20	12/18/20
3	75	Caucasian	M	Low energy	101	88	96	10/26/20	11/1/20	10/15/20	10/30/20
4	66	Caucasian	F	Loss of appetite, cough, chills, SOB	101	97	96	10/26/20	10/29/20	10/15/20	10/30/20
5	66	Caucasian	F	Vomiting, weak, body aches, anosmia	101	89	95	12/18/20	12/22/20	12/18/20	NA
6	43	Caucasian	F	PE, headache, body ache, cough	101	88	94	1/26/21	2/12/21	1/26/21	2/9/21
7	62	Caucasian	M	Productive cough, headache	102	86.5	91	11/24/20	12/8/20	11/13/20	12/8/20
8	57	Caucasian	M	Cough, nasal congestion, SOB, body aches	102	88	96	10/27/20	11/10/20	10/26/20	11/15/20
9	94	Hispanic	F	Low energy, SOB, confusion, loss of appetite, shaking	102	88	94	1/10/21	1/20/21	12/22/20	NA
10	66	Hispanic	M	Cough, SOB, respiratory failure	100.6	72	87	Declined	Death	12/22/20	NA
11	63	Hispanic	F	Cough, SOB	102	90	96	1/10/21	1/20/21	12/22/20	NA
12	47	Hispanic	M	SOB	104	84	91	12/19/20	12/25/20	12/16/20	NA
13	69	Caucasian	F	Cough, congestion, rash	102	88	91	11/17/20	12/3/20	11/13/20	NA
14	69	Caucasian	M	Post-nasal drip, cough, sinus pain	98	88	91	11/17/20	12/3/20	11/13/20	NA
15	71	Hispanic	M	Low energy, productive cough, anosmia	101	88	NA	12/17/20	1/5/21	12/13/20	NA
16	67	Hispanic	F	Dry cough, body aches, low energy, anosmia	100	88	NA	12/17/20	1/5/21	12/13/20	NA
17	46	Caucasian	F	Diarrhea, rash, renal pain	102	87	94	8/8/20	8/19/20	7/2/20	NA
18	86	Caucasian	M	Cough, fever, low energy	102	88	95	1/9/21	1/19/21	1/8/21	1/19/21
19	59	Caucasian	F	Stomach pain, diarrhea, cough, rash	102	90	95	9/16/20	9/25/20	8/19/20	NA
20	54	Muslim	M	Cough, fever, loss of appetite, chills	101.2	88	NA	10/16/20	10/28/20	10/15/20	10/28/20
21	92	Caucasian	M	Low energy	102	85	91	2/5/21	2/11/21	2/2/21	2/15/21
22	63	Hispanic	M	Cough, low energy, loss of appetite	101.3	90	96	2/2/21	2/12/21	2/2/21	NA
23	57	Hispanic	M	Cough, SOB	98	73	90	1/6/21	2/8/21	12/30/20	1/24/21
24	46	Hispanic	F	Chest pain, SOB	98.6	90	NA	2/18/21	2/24/21	2/17/21	NA
25	87	Hispanic	M	Severe SOB, low energy, trouble walking	101.6	90	95	2/27/21	3/5/21	2/17/21	NA
26	86	Caucasian	M	SOB	102	88	NA	Declined	Death	10/6/20	NA

ID: Identification number; NA: Not available; neg.: Negative; O_2_% sat.: Oxygen saturation just before time of treatment initiation; O_2_% sat. post 24 h: Oxygen saturation 24 h after treatment initiation; PE: Pulmonary embolism; pos: Positive; Rx start date: Day 1 of IVM Combination Therapy administration; SOB: Shortness of breath; Temp.: Temperature.

Given the dates of the study, it is very unlikely any subjects had the Delta or Omicron variant of COVID-19. Six subjects had their strains identified (data not shown) and were found not to have these variants.

Table 2 summarizes the demographics and past medical history (PMH) of subjects who consented to treatment (total n = 24; two additional subjects who declined treatment are excluded). Notably, patients were older (a known COVID-19 vulnerability), with a mean age of 66 ± 2.75 years old and a range of 43–94 years (Table 2A). The population of the 24 subjects consenting to treatment (not subjects #10 and #26, Table 1) was 63% males. Death of untreated subjects #10 and #26 excluded downstream analysis in the other figures.

**Table 2.** Demographics and clinical characteristics of subjects.

Age and demographics of subjects		
Age (mean, SEM, range)	66, 2.75, 43–94	
Male, n (%)	15 (62.5)	
Female, n (%)	9 (37.5)	
Race, n (%)		
– Caucasian	14 (58)	
– Hispanic Mexican	7 (27)	
– South American	2 (8)	
– Other	1 (4)	

Prevalence of COVID susceptible comorbidities		
Comorbidity	**Subjects (n)**	**Subjects (%)**
Type 2 diabetes mellitus	6	25.00
Heart or cardiovascular	5	20.83
COPD	3	12.50
Obesity (BMI 30–40)	3	12.50
Severe obesity (BMI ≥40)	2	8.33
Chronic kidney disease	1	4.17
Immunocompromised state	1	4.17

Concurrent comorbidities in subjects (n)		
**Comorbidities (n)**	**Subjects (n)**	**Subjects (%)**
0	13	54.17
1	6	25.00
2	3	12.50
3	2	8.33

COPD: Chronic obstructive pulmonary disease; SEM: Standard error of the mean.

Table 2B lists the number of patients who had comorbidities associated with COVID-19 vulnerability, based on CDC guidelines [21]. These comorbidities are chronic kidney disease, COPD, Down syndrome, cardiovascular disease, immunocompromised state (including HIV), obesity (BMI of 30 kg/m^2^ or higher but <40 kg/m^2^), severe obesity (BMI ≥40 kg/m^2^), pregnancy, sickle cell disease, smoking and Type 2 diabetes. Of note, no subjects had cancer, Down syndrome or sickle cell disease and none were pregnant or were smokers.

Many subjects had multiple comorbidities associated with COVID-19 vulnerability, as outlined in Table 2B. In total, 11/24 (45.83%) subjects had COVID-19-vulnerable comorbidities, of which three (12.50%) had two separate comorbidities and two (8.33%) had three comorbidities.

A minority of subjects (n = 7) had other COVID-19 treatment(s) prior to and/or during ICT administration, namely remdesivir (n = 1 subject); involvement in a placebo-controlled trial of hydroxychloroquine, azithromycin, vitamin D, zinc pack (HAZDpaC) (n = 4 subjects, trial clinicaltrial.gov NCT04334512; may have been given treatment or placebo); and hydroxychloroquine (HCQ) (n = 3 subjects).

Figure 1 demonstrates that all subjects recovered from COVID-19, typically within 1 to 2 weeks. Figure 1A shows various durations for each subject and average values (one outlier excluded). Time from onset of symptoms to treatment initiation is shown in column 1 and averaged 9.2 ± 2.1 days. The time from start of treatment to symptom resolution was 11.6 ± 1.4 days. Time from first positive to first negative PCR was 16.9 ± 1.6 days and was less than 3 weeks. The time from start of treatment to first negative PCR was 11.5 ± 1.6 days and was also less than 3 weeks.

**Figure 1.** Complete recovery was seen in all patients within 1 to 3 weeks. **(A)** Time in days to various stages of symptom onset and resolution. Nearly all subjects resolved symptoms and became PCR negative in 3 weeks. Col 1: Symptom onset to start of treatment (n = 23; mean: 9.17 ± 2.05). Col 2: Start of treatment to resolution of symptoms (n = 23; mean: 11.61 ± 1.38). Col 3: First PCR positive to first PCR negative (n = 10; mean: 16.90 ± 1.58). Col 4: Start of treatment to first PCR negative (n = 10; mean: 11.50 ± 1.60). **(B)** Top, 100% survival rate was seen in patients, which is significantly higher (p = 0.044 via Chi-Square, *χ*^2^, test) than synthetic control from CDC database of equivalent or less COVID-vulnerable subjects. Bottom, no (0%) patients required hospitalization, which is significantly less (p = 0.0011 via *χ*^2^ test) than synthetic control from database.

Figure 1B shows that 100% of subjects survived COVID-19, without the need for hospitalization or ventilator use. As noted in Table 2, many of these subjects were older and with comorbidities. When compared with the CDC synthetic control arm (see methods and as follows), this was a significant increase in survival rate (p = 0.044) and decrease in hospitalization rate (p = 0.0011), evaluated via χ^2^ test. Of note, the patients in the CDC database likely received treatment of an unknown nature. Thus, the survival rate of this synthetic control reflects the “typical” survival rate in the USA, which is significantly less than the 100% survival rate observed on ICT.

The 100% survival rate on ICT was compared with survival rates from the CDC database of COVID-19 subjects; 313,805 control subjects were obtained, based on the qualification criteria described in the methods section. These criteria focused on older subjects (50+ years of age), similar to the authors' population, who also had underlying conditions. One should note that the underlying condition criteria information available in this database refers to chronic conditions of any type, whether or not the condition induces COVID-19 vulnerability. With this definition, 100% of control subjects and ICT-treated subjects had underlying conditions of any type.

The critical finding in Figure 2 (see also Table 2) showed that 23/24 patients were hypoxic with SpO_2_ < 90%. Some subjects consenting to treatment had SpO_2_ as low as 73%, 77%, 84% and 85% on presentation. Figure 2A shows that the SpO_2_ of subjects was significantly less than 95%, the defined point of cure (95% CI of mean SpO_2_: 85.5% to 89.4%; mean: 87.4% ± 0.93). Subjects' SpO_2_ increased within 24 h of treatment. Their mean SpO_2_ before treatment (for subjects with data before and after 24 h) was 86.5% ± 1.3, and after 24 h of treatment 93.1% ± 0.63, a highly significant and rapid increase (p < 0.001). SpO_2_ then continued to rise. Treatment continued for 10 days reaching the point of successful treatment or cure, with SpO_2_ > 95%. Successful treatment was reached for all subjects. That is, there was a 100% restoration rate in terms of SpO_2_. No patient who accepted treatment required hospitalization.

**Figure 2.** All subjects reached successful treatment (SpO2 above 95%) and experienced significant increase in SpO2 within 24 h. **(A)** O_2_ saturation prior to treatment was significantly (p < 0.05) less than 95%, the defined successful treatment reached by all subjects. **(B)** O_2_ saturation significantly increased in subjects 24 h after treatment (paired *t*-test, p < 0.001, only subjects with data before and after treatment included). O_2_ saturation continued to rise until the defined cure of greater than 95% O_2_ saturation was reached.

Two subjects (#10 and #26) declined treatment. These subjects did not recover SpO_2_ and died from COVID-19 infection. An adverse drug event of dizziness was reported by one treatment subject who nevertheless continued with treatment successfully otherwise.

Figure 3 shows the validation of the Covidex and Covidex-F scores the authors developed, defined in the methods. These scores provide an index of COVID-19 predicted severity, based on PMH, O_2_ just before treatment and fever grade on presentation. The mean Covidex score was 10.34 ± 1.08 and the mean Covidex-F score was 11.63 ± 1.13, with 87% and 85% of the score points, respectively, coming from the contribution of the SpO_2_ term. In other words, approximately 80–90% of this score is weighted toward SpO_2_. It should also be noted that the PMH aspects that contribute to this score emphasize respiratory, cardiovascular and obesity histories and differ from CDC-defined COVID-19 vulnerabilities.

**Figure 3.** Ambulatory COVID scores, Covidex and Covidex-F (see methods for definition; Covidex-F includes fever measure) versus time from start of treatment to symptom resolution. There was a significant relation between either Covidex score (Covidex: p = 0.0288; Covidex-F: p = 0.0096) and treatment resolution time.

Covidex and Covidex-F are both plotted versus time from treatment to symptom resolution. Both show statistically significant correlations (Covidex: p = 0.0096, *r*^2^ = 0.2078; Covidex-F: p = 0.0288, *r*^2^ = 0.2790), indicating that either Covidex or Covidex-F is associated with and may predict time to symptom resolution.

## Discussion

The authors report for the first time a highly effective outpatient ICT, which prevented hospitalization and led to 100% survival and cure in unselected ambulatory ‘moderately to severely’ ill COVID-19 patients with hypoxia. Given the authors' experience developing combination therapies for *H. pylori*, they clinically explored (without formal comparative studies) several different IVM-based combinations on ambulatory COVID-19 patients, searching for a cure, and found the above combination to be very effective as a therapy for COVID-19. Some patients needed a personalized medicine approach, using HCQ or other components, much the way *H. pylori* resistant to triple therapy sometimes requires quadruple therapy. The authors acknowledge that they did not have the capacity in this study to test every permutation of ingredients with a scientific trial, yet such studies can be useful for future refinement. Applying IVM via weight-based dosing has been suggested [22], but more importantly, appropriate doses may be needed to cover various COVID-19 strains.

Hypoxia is a demonstrated predictor of COVID-19 mortality. For example, several of these patients had profound hypoxia, measured by oximetry at 73%, 77%, 84% and 85% on presentation. Despite a symptom to treatment delay of 9.2 days, this treatment brought rapid improvement – beginning in some within 12 h with a mean SpO_2_ rising from 86.5 to 93.1 in the first 24 h. There was a parallel improvement in the symptoms, including loss of cough, fever and tiredness. Also, the time from the start of treatment to the first negative PCR averaged 11.5 ± 1.6 days. Generally, such ill patients would have been admitted to the hospital, yet all those treated with ICT avoided hospitalization and none died.

Turning to the ECT ‘synthetic control arm’, it is clear that ICT was statistically superior to the control arm, even though a small patient group was reported. The very low number of adverse effects from reported studies and this treatment group support the use of ICT if clinical symptoms and risk factors for COVID-19 progression are present, even in cases with PCR pending results. ECT arms are now increasingly used, especially where the control arm or ‘standard-of-care’ arm may have a fatal outcome [23].

The rationale for exploring a combination antiviral therapy approach is based on our growing understanding that intracellular infections – bacterial or viral – generally cannot be cured using a single drug. Multiple drugs address numerous mechanisms of viral replication and can cure multiple strains. Even therapies using two drugs, such as two antibiotics for *H. pylori*, have resulted in resistance. Multiple-drug therapies, especially using three or more, are expected to be more effective at reducing viral load, thereby limiting resistance and variant development [24], as reviewed for HIV [18]. Use of IVM alone, on the other hand, has already led to resistance when treating scabies, nematodes, strongyloidiasis, microfilaridermias and *Onchocerca volvulu*s [17,25–28]. All these diseases are based on eukaryotic organism infection, not viral, and are thus far less prone to mutations and consequently resistance. Since IVM resistance has occurred on occasion for these diseases and since COVID-19 has become a pandemic, resistance needs to be proactively prevented for COVID-19 and its future variants. Given the current state of the pandemic, we cannot permit IVM resistance to develop clinically, and be experimentally demonstrated, before it is addressed. Thus, IVM in COVID-19 should not be used as a monotherapy, only in combination therapies, especially so with growing reports of mutant strains resulting in vaccine breakthrough infections. Combination therapy could allow for more rapid cures, resistance prevention and overcoming of mutant strain emergence – ‘no replication, no mutation’.

Regarding strategies in the development of combination therapies, intracellular coronavirus replication requires several active drugs to inhibit viral replication. IVM, doxycycline and zinc all individually inhibit coronavirus replication and, although there are other candidates, the authors have proposed the above combination based on its efficacy, component safety profiles, inexpensive nature and lack of drug–drug interaction. The combination of IVM and doxycycline has been shown to be somewhat effective for COVID-19 [7], potentially (statistical trend) more effective than the HCQ and azithromycin combination [29], and mechanistically theorized as synergistic [30], even though doxycycline alone is not considered effective [31]. Further, given that zinc plays a key role in antiviral activity [32,33], it would combine well with the ionophores (IVM and doxycycline) to increase its intracellular concentration and expedite viral clearance [34]. Also, the combination of zinc with IVM and doxycycline has no reported drug–drug interactions [35]. Additionally, each of these drugs has a low adverse side-effect profile and no QT prolongation as reported with azithromycin [22,36–38].

Overall, based on the current literature, a 10-day combination therapy of IVM, doxycycline and zinc will not only improve symptoms [6,7] but also accelerate recovery from COVID-19. The authors have chosen a safe IVM dosage, approved for parasites, of 36 mg over 10 days, and this dose has been shown to be both effective and safe in COVID-19 treatments [39]. The staggered IVM dosage over 10 days is proposed based on the half-life clearance of the drug in plasma (up to 66 h) [40]. The proposed duration would allow constant availability of adequate plasma level IVM to facilitate zinc entry into the cells. Hence, the above rationale explains why some publications have already shown that IVM alone is not adequate to cure COVID-19, while a multidrug regimen is likely to be more efficacious [41].

This study enrolled consecutive subjects (i.e., as subjects presented, they were enrolled and none were turned down) in the study and did not bias subject selection from different time points. Many of the enrolled subjects were profoundly ill with subjective assessments that may have resulted in hospital admission and/or intubation, yet ICT activity appears to have rapidly restored SpO_2_ and reversed other symptoms, which could not be explained simply by the developing immunity. The authors acknowledge that a major limitation of the study is the small sample size (n = 24 consenting to treatment) in this preliminary study, which may limit its generalizability. These subjects consisted of the first set to present to Ventura Clinical Trials, and more data are being collected. Of note, many such severely ill patients may not opt for the unknown of a less established clinical trial for a serious case of COVID-19. The authors' future studies will expand the sample size, test the effect of other IVM dosages and explore the mechanistic contribution of the microbiome to IVM's effectiveness in COVID-19.

While a concomitantly enrolled control arm would be ideal for a true RCT, this is not feasible with severe COVID-19. Given the potentially fatal outcomes, Lawrie *et al.* [42] said, “*Placebo-controlled trials of ivermectin treatment among people with COVID-19 infection are no longer ethical and active placebo-controlled trials should be closed*,” the effects of which observed in the two subjects who declined treatment and did not survive. Hence, this study has made use of the ECT or ‘synthetic’ control arm [23], which has enabled the authors to make matched age and comorbidity comparisons. Institutional review boards should now include a provision to allow for synthetic arm studies and reject COVID-19 trials that utilize a control arm as published by Lawrie.

## Conclusion

This study builds on extensive literature to provide practical, inexpensive, safe, readily available and highly effective IVM triple therapy aiming to prevent resistance and one that can confidently be used as a routine treatment for outpatient COVID-19.

**Summary points**

- The authors observed the effectiveness of a novel combination of ivermectin, doxycycline, zinc and vitamins D and C in 24 COVID-positive subjects with high-risk features/comorbidities.
- The majority of the subjects were hypoxic (23 out of 24; oxygen saturation [SpO_2_] <90%), with 4 below SpO_2_ <85% on presentation. Many subjects had related comorbidities (n = 11; 45.8%). The median age of all subjects was 66 years old.
- Intervention consisted of 10 days of doxycycline (100 mg twice a day), ivermectin (12 mg on day 1, day 4 and day 8), zinc (25 mg twice a day), vitamin D3 (1500 IU twice a day) and vitamin C (1500 mg twice a day). All treatment was given orally and ceased at the end of 10 days.
- One hundred percent of patients accepting treatment survived without the need for hospitalization. All subjects recovered from hypoxic symptoms (SpO_2_ >95%) within 10 days of treatment.
- The authors report an effective and inexpensive COVID therapy preventing hospitalization and death in all patients and rapid resolution of hypoxia in these ambulatory ‘moderately to severely’ ill patients.
